# Epidemiological Study of Lung Cancer and Clinical Medication in England from 2001 to 2019

This article has been retracted.

**DOI:** 10.1155/2022/3577312

**Published:** 2022-03-23

**Authors:** Baokun Zhang, Ying Yang

**Affiliations:** The University of Sheffield, Western Bank, Sheffield S10 2TN, UK

## Abstract

We aimed to explore the epidemiological characteristics and changes of lung cancer and the clinical medication in England from 2001 to 2019. We searched related research using search engine systems such as MEDLINE, PubMed, and PsychINFO. Lung cancer is a serious disease and the prognosis is usually very poor. The overall mortality rate of lung cancer decreased year by year in England from 2001 to 2019, but men, the elderly, and people exposed to polluted air are still more likely to be infected with lung cancer or die as a result, the prevalence and mortality rate of lung cancer in the north of England is significantly higher than that in the south, and the gap is increasing year by year. Lung cancer has changeable risk factors such as quitting smoking and improving air quality, which can effectively reduce the related risk. Paclitaxel, docetaxel, gemcitabine, and vinorelbine are the main drugs for the treatment of lung cancer in England and the treatment of these drugs is beneficial to the survival and quality of life of patients. Men and the elderly are at high risk of lung cancer, which means that lung cancer has obvious gender inequality and age inequality. At the same time, based on the statistical data of lung cancer risk in different regions, it can be concluded that lung cancer also has strong geographical and economic inequality. Changing risk factors and using drugs can effectively reduce the risk of lung cancer and provide effective treatment.

## 1. Introduction

Lung cancer is a serious threat to human health [1]. According to the results of WHO statistics from 2001 to 2019, lung cancer ranks among the top ten causes of death in the world every year (https://www.who.int/news-room/fact-sheets/detail/the-top-10-causes-of-death). In the UK (England, Wales, and Scotland**)**, about 35000 people die from lung cancer each year and lung cancer is still the leading cause of death in England today [2]. According to statistics from Figure 1 (https://ec.europa.eu/eurostat/en/web/products-eurostat-news/-/edn-20180531-1), for the UK, lung cancer accounted for 22% of all cancers reported in 2015. This ranks eighth among all countries and the percentage is higher than the average of European countries (22% vs 21%). This shows that lung cancer is a very serious public health problem in England in recent years, which has seriously affected the health and life expectancy of many people; because the proportion of people with lung cancer in England is very high and a large number of people die of lung cancer every year, it should be paid enough attention to by people in England.

## 2. Epidemiology

Lung cancer can start anywhere in the lungs or respiratory tract. It is also a disease caused by many factors, such as smoking, air pollution, and other lung diseases. It is the deadliest cancer in the world [3]. The main symptoms of early patients often have symptoms such as coughing and chest pain. Once patients have typical clinical manifestations such as hemoptysis, most of them are in the middle and late stage. When lung cancer enters the middle and late stage, most patients have lost the opportunity of operation, so lung cancer is easy to be ignored in the early stage, but the survival rate is very low when it is found in the later stage. At present, the treatment of lung cancer includes surgical treatment and chemotherapy, but the prognosis is usually very poor [4], so it is particularly important to prevent the occurrence of lung cancer by changing risk factors.

For England as a whole, it can be seen that from Figure 2 (https://fingertips.phe.org.uk/search/lung%20cancer#page/0/gid/1/pat/6/par/E12000004/ati/101/are/E07000032/iid/1203/age/1), from 2001 to 2019, although the mortality rate of lung cancer patients in England fluctuated slightly at adjacent time nodes, the overall trend of the value decreased (from a peak of 65.1/100,000 in 2001 to 53/100,000 in 2019). This shows that although lung cancer is still a fatal disease in England, the overall mortality rate of patients with lung cancer is still declining steadily by 2019. The data uses direct standardized rate. The directly standardized rate is an important tool for showing a highly age-dependent disease, such as cancer [5]. The unit is 100,000 people, and the standard population is the 2013 European standard population.

The definition of mortality of lung cancer is the age-standardized rate of mortality from lung cancer in persons of all ages per 100,000 population, the source of the data is Public Health England based on ONS source data. The significance of the age-standardised rate of mortality is to allow researchers to compare the statistical data directly with each other, because only by using such a general standard can the population and number of people of different ages be discussed at the same time. According to Figure 3, it can be seen that the mortality rate of lung cancer has a great difference for gender. Statistics from 2017 to 2019 shows that the mortality rate of females is 44.6/100,000, while men is as high as 63.6/100,000, and there is about 30% difference between men and women. This is because men have higher smoking rates than women in England, and men are also more likely to develop lung cancer [6]. At the same time, lung cancer becomes more common with age, about 45% of lung cancer patients in England are older than 75 years old, and for the acceptance rate of lung cancer treated by related surgery, the acceptance rate decreases sharply after the age of 75, and the acceptance rate at the age of 80 is half of that at the age of 70 (https://www.cancerresearchuk.org/about-cancer/lung-cancer). It shows that men have a higher prevalence of lung cancer and have worse living conditions than women and older people are also more vulnerable to lung cancer.

The distribution of morbidity and mortality of patients with lung cancer is characteristic in different parts of England. First, studies have shown that the incidence of lung cancer in the north of England is higher than that in the south [6]. The color distribution in Figure 4 shows that from 2017 to 2019, most of the red and yellow areas are concentrated in the north part, while the south is dominated by green, which means that the mortality rate of lung cancer in the north is higher than that in the south. The main cause of the phenomenon is economic inequality. Study of Arik et al. showed that the incidence of lung cancer is high in poor areas of England and the number of the poor in the north is higher than that in the south. This is consistent with the conclusion that the incidence of lung cancer is high in the north. When poor people have lung cancer, they have limited funds for treatment, which leads to an increase in mortality, and this geographical difference is increasing year by year [6]. The evidence suggests that people living in the north of England have higher rates of lung cancer and mortality, while the poor are more vulnerable.

## 3. Modifiable and Nonmodifiable Risk Factors

First, smoking is one of the most important risk behaviors of lung cancer and a large number of studies have found that smokers have a 15–30 times higher risk of developing lung cancer than nonsmokers [4]. So, smoking has a profound impact on the prevalence of lung cancer, but quitting smoking is a changeable behavior for people to reduce the risk of lung cancer. Studies have shown that people who quit smoking at the age of 22 have a relative risk of dying from lung cancer in the future compared with those who have never smoked which is 1.56 (95% Cl: 1.03–2.37), and those who quit smoking at 45–55 have a relative risk of dying from lung cancer compared with those who have never smoked 5.91 (95% Cl: 5.01–6.97) [7]. The meaning of the confidence interval (Cl) is that it is a range of values used to quantify the inaccuracy of estimating a particular indicator. 95% Cl means that if you sample 100 times, you can get 100 confidence intervals, then at least 95 confidence intervals contain the overall mean. It can be seen that quitting smoking earlier can greatly decrease the risk of lung cancer. Air pollution can also lead to an increased risk of lung cancer, including air pollution in residential homes and occupational exposure. A study in England showed that the relative risk of lung cancer increased by 0.08 (95% Cl: 0.03–0.20)/100 Bq M^−3^ increase in the observed time-weighted residential radon concentration [8]. Another study shows that asbestos is an important risk factor for lung cancer and if full exposure to asbestos for one year or moderate exposure for 5–10 years can double the lung cancer risk, 7 to 15 years after cessation of asbestos exposure, the risk of lung cancer may be reduced or disappeared [9]. This shows that although smoking and air pollution can increase the risk of lung cancer, it can be reduced by quitting smoking, long hours of massive ventilation, and protective measures at work.

There are other factors that affect the incidence and mortality of lung cancer, such as genetic and previous lung diseases like COPD. The susceptibility to lung cancer is partly caused by individual genes [10]. This means that some people are inherently more likely to have lung cancer, and there is no way to change the genes, so this part of risk cannot be removed. Epidemiological studies have shown that COPD can increase the risk of lung cancer by 4–6 times [11]. It shows that once you have had a disease like COPD, the risk of life-long suffer from lung cancer will be greatly increased, and there is still no way to reduce this risk.

## 4. Clinical Medication

Paclitaxel, docetaxel, gemcitabine, and vinorelbine are the main drugs for the treatment of lung cancer in England. The treatment of these drugs is beneficial to the survival and quality of life of patients, especially when used as combination therapy. Although the improvement in their median survival time is only 2 to 4 months, the effect is considerable in view of the fact that the survival time of untreated patients is often only about 5 months [12]. In addition, it is important that these survival rates are not improved at the expense of the patient's quality of life, and the quality of life is improved to some extent compared with BSC or older chemotherapy drugs. The term BSC is used to describe care which includes relief of symptoms by, for example, analgesics, but which does not attempt to prolong life or to remove the cause of the symptoms. BSC may vary in its inclusions [12]. First of all, the median survival time of patients treated with paclitaxel was significantly improved compared with BSC (4.8 months, 95% CI: 3.7 to 6.8, *P* < 0.05), which was of great help to prolong the lifespan of patients [13]. Docetaxel as a first-line treatment had limited effect on patients' overall health and physical function, but significantly improved emotional function, nausea/vomiting, pain (*P* < 0.0001), and dyspnea (*P* < 0.05); when used as second-line therapy, docetaxel had a significant beneficial effect on pain relief (*P* < 0.01) [14]. However, patients who received docetaxel had a higher frequency of hematological toxic events than those treated with BSC [12]. The incidence of continuous improvement of quality of life in patients treated with gemcitabine and BSC was significantly higher than that in patients treated with BSC alone (22% vs. 9%, *P* < 0.005), and chest pain was significantly improved in patients treated with gemcitabine (*P* < 0.005) [15]. At the same time, there was no significant difference in adverse reactions between patients treated with gemcitabine and other drugs and methods [12]. The median survival time of patients treated with vinorelbine was improved and there were significant improvements in cognitive function (*P* < 0.05), dyspnea (*P* < 0.05), and painkillers (*P* < 0.01) [16]. But, the adverse reactions also included constipation, leukopenia, neutropenia, vomiting, and hair loss [12].

## 5. Critical Discussion of Study Results

There are strong geographical differences in the prevalence and mortality of lung cancer, which is also the focus of people's research. The study of Jack et al. in 2003 explored the treatment and geographical differences in the survival of lung cancer patients in England [17]. Although the use of retrospective studies can bring the findings closer to reality, more issues should be discussed when conducting in-depth studies.

The study used a large sample of 32818 patients from The Thames Cancer Registry who had previously been diagnosed with lung cancer, and while the use of this database can guarantee the quality of the data, there should be a lot of potential criticism.

First, although these patients have lung cancer, they do not have statistics on whether they have other diseases, because mortality and life expectancy are affected by other diseases. The study's failure to count such data can lead to avoidable deviations such as deviations in the one-year and three-year net survival rates of these patients. Secondly, for these patients, they only pay attention to the means and location of treatment, but do not pay more attention to their daily living conditions, such as smoking and alcohol abuse, which are easy to aggravate the illness and cause other illnesses. According to the research, patients who actively treat and choose to see a doctor in the radiotherapy center for the first time have a longer survival time, but the specific length of life is also related to the lifestyle during the treatment period. Therefore, the experiment does not have better control variables in this respect.

The authors conclude that there are geographical inequalities in the treatment and survival of lung cancer patients in East England, for example, these inequalities may be caused by different access to oncology services, but for future related research, it can pay more attention to the impact of local policies and their changes on the survival rate of different regions, such as local medical security policies, which are also lacking in the research of their study.

## 6. Conclusion

Lung cancer is a serious disease. The overall mortality rate of lung cancer decreased year by year in England from 2001 to 2019, but men, the elderly, and people exposed to polluted air are still more likely to be infected with lung cancer or die as a result, the prevalence and mortality rate of lung cancer in the north of England is significantly higher than that in the south, and the gap is increasing year by year. Lung cancer has changeable risk factors such as quitting smoking and improving air quality, which can effectively reduce the related risk, and paclitaxel, docetaxel, gemcitabine, and vinorelbine help patients with lung cancer and can improve their quality of life to some extent.

## Figures and Tables

**Figure 1:** Share of lung cancer in all cases of fatal cancer in the EU member states, 2015.

**Figure 2:** Mortality rate form lung cancer for England (public health England 2020).

**Figure 3:** Mortality rate from lung cancer in England.

**Figure 4:** Map of district in England for mortality rate from lung cancer (directly standardized rate per 100,000, 2017–2019).

## Data Availability

The datasets used and analyzed during the current study are available from the corresponding author on reasonable request.
